The article "Altered Structural and Functional Abnormalities of Hippocampus in Classical Trigeminal Neuralgia: A Combination of DTI and fMRI Study" was published in 2022. Journal: J Healthc Eng.

# Altered Structural and Functional Abnormalities of Hippocampus in Classical Trigeminal Neuralgia: A Combination of DTI and fMRI Study

**DOI:** 10.1155/2022/8538700

**Published:** 2022-11-30

**Authors:** Yongming Tan, Chun Zhou, Laichang He

**Affiliations:** The First Affiliated Hospital of Nanchang University, Department of Radiology, Yong Wai Street 17, Nanchang, Jiangxi 330006, China

## Abstract

**Purpose:**

Diffusion tensor imaging (DTI) and resting-state functional magnetic resonance imaging (rs-fMRI) were applied to speculate the altered structural and functional abnormalities within the hippocampus in classical trigeminal neuralgia (CTN) patients by detecting the alteration of apparent diffusion coefficient (ADC), fractional anisotropy (FA), and regional homogeneity (ReHo). *Patients and Methods*. Multimodal MRI dataset (DTI and fMRI) and clinical indices (pain and neuropsychological scores) were collected in 27 CTN patients and 27 age- and gender-matched healthy controls (HC). Two independent-sample *t*-tests were performed to compare the ADC, FA, and ReHo values in hippocampus areas between CTN patients and HC. Correlation analyses were applied between all the DTI and fMRI parameters within the hippocampus and the VAS (visual analog scale), MoCA (Montreal cognitive assessment), and CDR (clinical dementia rating) scores.

**Results:**

CTN patients showed a significantly increased FA values in the right hippocampus (*t* = 2.387, *P* = 0.021) and increased ReHo values in the right hippocampus head (voxel *P* < 0.001, cluster *P* < 0.05, FDR correction) compared with HC. A positively significant correlation was observed between the ReHo values and MOCA scores in the right hippocampus head; FA values were also positively correlated with MOCA scores in the right hippocampus.

**Conclusion:**

CTN patients demonstrated an abnormality of structures and functions in the hippocampus, which may help to provide novel insights into the neuropathologic change related to the pain-related dysfunction of CTN.

## 1. Introduction

CTN is characterized by unilateral facial pain with an abrupt onset and offset, which localizes to one or more branches of the trigeminal nerve [1]. It is generally considered that the most common cause of trigeminal neuralgia is the compression of trigeminal nerve by vessels, especially the arteries [2, 3]. Suffering from severe facial pain, CTN patients not only present significant social disability [4] but also present cognitive decline, memory loss, anxiety, depressive tendencies, and negative pain-related changes [5]. The latest research related to CTN shows that the central nervous system (CNS) plays a major role in the regulation and maintenance of pain [6–8]. Chronic pain can cause structural and functional abnormalities in pain-related networks and trigger functional reorganization, including those involving hippocampus [9]. Hippocampal is an important part of the limbic system, which is usually considered as an organ that produces memory and emotions. Although previous studies have also described the involvement of hippocampal circuits in pain treatment and neurogenesis regulation in animal models of chronic pain [10], the relationship between the hippocampus and chronic pain in CTN patients has not been clearly defined. Diffusion tensor imaging (DTI) studies have found that the white matter has a reduced FA value associated with the course or symptoms of patients with chronic pain, such as migraine or temporomandibular disorder pain [11]. Similarly, spatial statistical analysis based on the white matter skeleton confirmed that FA reduction in CTN patients mainly occurred in the corpus callosum, cingulate, posterior, and longitudinal bundles. This damaged white matter mainly involved the fiber bundles connecting to brain functional areas such as sensation, cognition, emotional dimensions, and attention [12]. These microstructural abnormalities of the CTN may be related to pain conduction and regulation imbalance in the central nervous system. However, there is still no clear research on whether there is a microstructure abnormality in the hippocampus of CTN patients.

The article "Altered Structural and Functional Abnormalities of Hippocampus in Classical Trigeminal Neuralgia: A Combination of DTI and fMRI Study" was published in 2022. Journal: J Healthc Eng.

Resting-state fMRI is an alternative method to measure spontaneous activity of brain. At present, several key brain regions of the CTN have been revealed, including the default mode network, saliency network, and sensory-motor network [13–15]. These areas are closely linked to pain perception, regulation, cognitive-emotional interaction, and motor control, but there are few fMRI studies on the hippocampus of the CTN. Regional homogeneity (ReHo) reflects the oscillation synchronicity of intraregional cortical neurons (an important aspect of resting-state spontaneous neuron activity), which has been reported as a basic mechanism of neuron function. Abnormal ReHo may be related to changes in the temporal spontaneous neural activity of a certain region, and ReHo may provide information that is critical to fully understanding CTN-related functional brain alterations [16]. DTI can reveal microstructure alterations of the brain. Combined with these methods, we hypothesized that the microstructure and function of the CTN hippocampus were abnormal. In this study, the hippocampus was taken as the ROI. ReHo and DTI were used to analyze the possible abnormal changes of hippocampal microstructure and function in CTN patients and explore the effects of these abnormalities on cognitive function, memory, and emotion.

The article "Altered Structural and Functional Abnormalities of Hippocampus in Classical Trigeminal Neuralgia: A Combination of DTI and fMRI Study" was published in 2022. Journal: J Healthc Eng.

## 2. Materials and Methods

### 2.1. Patient Population

From April 2017 to March 2018, a total of 27 CTN patients were recruited. In the meanwhile, 27 healthy controls (age-, gender-, and education level-matched) were included in this study for HC. The inclusion criteria were based on the diagnostic criteria of the classic trigeminal neuralgia of the International Association of the Study of Pain (IASP) [17]. The exclusion criteria were as follows: (1) frequent spontaneous neuralgia (>25 times per day); (2) atypical neuralgia; and (3) under treating neuralgia. All of them had no MR contraindications. Experiments were conducted with the written consent of each participant and were approved by the biomedical ethics committee of The First Affiliated Hospital of Nanchang University.

### 2.2. MRI Data Acquisition

The MRI data were acquired with a 3.0 T MR scanner (Siemens, Erlangen, Germany). The subjects were required to take it easy, close their eyes, keep awake, keep still, and think of nothing during the scan. The functional images were obtained using a gradient echo-planar imaging sequence. Parameters are as follows: TR/TE = 2000 ms/30 ms, flip angle = 90°, FOV = 200 × 200 mm, matrix resolution = 64 × 64, 30 sections, and gap = 1.5 mm, 2 mm slice thickness. High resolution three-dimensional T1-weighted anatomy data parameter: including entire brain, turbo field echo sequence, TR = 1900 ms, TE = 2.26 ms, flip angle = 9°, FOV = 240 × 240 mm, resolution = 256 × 256 matrix, slices = 176, thickness = 1 mm, voxel size = 1.0 × 1.0 × 1.0 mm^3^, and interslice gap = 0.5 mm. One hundred and seventy-six sagittal slices images were acquired. The DTI images were obtained axially 8 min 15 seconds using an echo-planar imaging sequence. Parameters are as follows: TR/TE = 7200 ms/104 ms, NEX = 1, FOV = 230 × 230 mm, matrix resolution = 128 × 128, 65 sections, gap = 2.5 mm, slice thickness with no gap, and 32 nonlinear dispersion gradients (*b* = 0, 1000 s/mm).

### 2.3. Functional Image Preprocessing and ReHo Analysis

As for fMRI and DTI data of left trigeminal neuralgia patients, the hippocampus image of the left trigeminal neuralgia patients was reversed to the right side of the sagittal plane via applying the NIFTY software package based on Matlab7.14 (R2012a) platform. So, the right side of all CTN patients is the affected side, and the left side is the unaffected side.

The fMRI data were preprocessed by applying the data processing assistant for resting-state fMRI Advanced Edition (DPARSFA) V2.3 running on Matlab7.0 1.3 (2012a) (Math Works, Natick, MA, USA). Remove the top 10 time points (excluding the influence of the environment). The corrected images were spatially normalized to a Montreal Neurological Institute template brain based on the standard stereotaxic coordinate system. Head motions were <1.5 mm most displacement in *z* direction and <1.5° in any directions. The low frequency signal drift was removed with a high-pass filter at 0.01∼0.1 Hz. that every voxel's time series was transformed into a frequency domain in order to gain the power spectrum. The square root at each frequency of the power spectrum was calculated and then obtained at 0.01–0.1 Hz at each voxel. Save the right hippocampus (automated anatomical label, AAL38) as a mask separately, then resample the right hippocampus by 3 × 3 × 3 mm. Kendall-w was calculated to measure ReHo or the local synchronization of the ranked time series within a functional voxel with the 27 nearest neighboring voxels. For standardization purposes, individual ReHo maps were divided by their global average within the right hippocampus mask. Then, spatial smoothing was performed using a 6-mm full-width-half-maximum Gaussian kernel. The procedures used to visualize the ReHo map results were implemented by using the resting-state fMRI Data Analysis Toolkit V1.8 (https://pub.restfmri.net).

The article "Altered Structural and Functional Abnormalities of Hippocampus in Classical Trigeminal Neuralgia: A Combination of DTI and fMRI Study" was published in 2022. Journal: J Healthc Eng.

### 2.4. Image Preprocessing: DTI Metrics

The diffusion tensor model is set for each voxel by using the FMRIB diffusion toolbox in FSL, and FA and ADC images are generated. That DTI data converted by MRIcroN software was input into the Diffusion Toolkit 0.6.4 (https://www.trackvis.org/) software for the FACT algorithm and reorganization parameter processing. Next, the resampled right hippocampus was spatially normalized and inverse transformed under statistical parametric mapping (SPM8) software. The relevant data obtained after each subject was processed by the Diffusion Toolkit software, then it was loaded into Track Vis 0.6.1. Next, the right hippocampus Mask (AAL38) was added, so the fractional anisotropy (FA) and apparent diffusion coefficient (ADC) values of each mask were recorded (Figure 1).

### 2.5. Statistical Analysis

Two independent-samples *t*-test was performed to compare the ADC and FA between CTN patients and HC by using the SPSS21.0 software. ReHo data in the hippocampus were analyzed by using statistical parameter mapping software between the CTN group and the HC. For all the above analyses, the significance level for the resultant statistical maps was set at <0.05. All ReHo data statistics are using the FDR-corrected (voxel *P* < 0.001, cluster *P* < 0.05) and the correction is limited within the hippocampus. DTI relative parameters and ReHo values in hippocampus were correlated with clinical variables by Pearson's linear correlation analysis under the SPSS software (*P* < 0.05).

The article "Altered Structural and Functional Abnormalities of Hippocampus in Classical Trigeminal Neuralgia: A Combination of DTI and fMRI Study" was published in 2022. Journal: J Healthc Eng.

## 3. Results

There was a significant difference between CTN patients and HC in VAS, MOCA, and CDR scores (Table 1).

The CTN patients show significant increases in ReHo in the right hippocampus head (MNI (3, −8, −27), peak intensity 3.7685, cluster voxels 14), in contrast to the HC (*P* < 0.05) (Figure 2). Moreover, compared to HC, the CTN patients also showed an increase in FA values in the right hippocampus (*P* < 0.05) (Table 2).

There was a positive significant correlation between the ReHo values, and MOCA scores in the right hippocampus head. FA values were positively correlated with MOCA scores in the right hippocampus (*P*=0.049) (Table 3). But we found no significant correlation between the ReHo values and the FA and ADC values (Table 4).

## 4. Discussion

Chronic pain triggers activity in a massive network of brain areas which was known as the “pain matrix,” including the primary (S1) and secondary (S2) somatosensory cortices, insula, anterior cingulate cortex (ACC), and the thalamus [16]. CTN is a typical case of chronic neuropathic pain. According to the study of Tracey [18], the mechanism of pain is not thought to result from the activation of one or more specific brain regions but from the emerging information interaction and influence among these regions. Noxious stimulations are transmitted from the peripheral nerves to the spinal cord by peripheral receptors, processed by the spinal cord, and transmitted through the medial and lateral conduction pathways [19]. The medial conduction pathway including thalamus and ACC, specifically conducts pain-related cognition and emotions [20]. Chronic pain may cause not only sensory dysfunction (spontaneous pain, hyperalgesia, and allodynia) but also various functional disorders, such as anxiety. These comorbidities of chronic pain make it necessary to extend the pain research from the lower levels of the “pain matrix” to the higher levels of cortical and subcortical brain structures. The hippocampus is composed of three parts: the hippocampus head, hippocampus body, and hippocampus tail. The hippocampus head is mainly folded in the CA1 area, which subserves episodic memory processes [21]. Cognitive impairment is observed in patients with pain [22]. A pain-induced decrease in hippocampus cell proliferation was recently confirmed by an immunoblotting study [23]. Accumulating evidence from animal and human studies suggest that the hippocampal formation may also bear significant associations with pain processing [24], Pain that becomes persistent or chronic pain, could produce profound effects on hippocampus anatomy, metabolism, morphology, and function [24]. ReHo abnormalities may reflect the abnormal local neuronal activity. A lower ReHo may represent local or intraregional reduced neuron activity or a regular disorder, which can strongly affect the brain neurons involved in information processing [16]. Enhanced ReHo reflects neuron activity in the region of the brain by increasing time synchronization and strengthening brain function. One reason why ReHo increased is the enhanced hippocampus activity synchronization by acute painful stimulation in the CTN [25]. In addition, the increasing of ReHo values in the hippocampus head may be a compensatory mechanism for the deficits of memory and pain-related emotion induced by painful stimulation in CTN patients.

The article "Altered Structural and Functional Abnormalities of Hippocampus in Classical Trigeminal Neuralgia: A Combination of DTI and fMRI Study" was published in 2022. Journal: J Healthc Eng.

It is well known that pain is a complex experience; not only does it depend on the regulation of sensory systems but also depends on the activation of mechanisms which control mood and affect emotional cognition in higher brain centers [26]. Until now, there has been some evidence suggesting that long-term plastic changes in sensory-related synapses are key mechanisms for chronic pain [27, 28]. Not only the changes in nerve fibers and synapses of the brain region associated with chronic pain are the necessary for regulation of chronic pain but also in multi-integrative brain structures during the experience and the anticipation of pain [29]. DTI, a brain imaging technique which is sensitive to the inherent diffusion of water molecules, can evaluate the hippocampus microstructure. ADC is a DTI metric that reflects the average dispersion of water molecules, affected by cell size and integrity. FA reflects the consistency of water molecules movement, associating with the destruction of microstructure and axon density or orientation [30]. It has been reported that structural alterations of the brain in the form of higher or lower gray matter density and volume and cortical thickness occur in a wide range of chronic pain conditions [9]. In this study, FA values in CTN patients were higher than HC, which indicates the increasing of the gray matter density or myelinated axon density in the hippocampus. It may be a compensatory change in the hippocampus under long-term stimulation from chronic pain. This result is consistent with the elevated ReHo prompting enhancement of hippocampus neuronal activity. However, there is no statistically significant difference in ADC values between CTN patients and HC. The possible reason is that the structural changes of the hippocampus in patients are not the result of destruction of hippocampus neurons, but rather the remodeling of synapses and myelinated nerve fibers. In addition, fractional anisotropy is less efficient than mean diffusivity for quantifying microstructural integrity as a microstructural index of hippocampus disease in the clinical context. The animal experiment results of Jackson and Regenstein [31] are in line with our results.

The article "Altered Structural and Functional Abnormalities of Hippocampus in Classical Trigeminal Neuralgia: A Combination of DTI and fMRI Study" was published in 2022. Journal: J Healthc Eng.

Now, there is a consensus that pain could cause not only sensory dysfunction but also miscellaneous functional brain shambles when it becomes persistent or chronic, such as anxiety, retrograde amnesia, agrypnia, and depression [32, 33]. Hippocampus is an integral component of the limbic system [34], which has been connected with some functions such as learning and memory [35], emotion and affect [36], and sensory-motor integration [37]. Intriguingly, a cortical-limbic pathway has been depicted to transit from S1 and S2 to the IC and parietal cortical structures, then to the amygdala, the perirhinal cortex, and the hippocampus. This pathway merges sensory pain features with information from other sensory systems, such as learning and memory, thus increasing a cognitive orientation regarding long-term results of affective pain processing [38]. In our research, there was a positive significant correlation between the ReHo/FA values and MOCA scores, which indicates a clear correlation between cognitive dysfunction and hippocampus function and structure dysfunction in CTN patients. Evidence from animal studies has suggested that neuropathic pain affects the learning and memory of rats, and its mechanism may be related to the decrease of P2X4 mRNA expression in hippocampus neurons [39]. There is a vast interaction between the systems involved in pain machining and other affective and motivational systems, and the hippocampus has extensive functional connections with the S1 and S2, the insula, the ACC, the thalamus, and so on [40]. Changes in the structure and function of the hippocampus in CTN patients may cause abnormalities in functional connections within the pain-related brain areas, which may result in depression and anxiety.

## 5. Conclusion

In summary, our research results show that ReHo and FA in the hippocampus of CTN have changed, which preliminarily proves the microstructure and functional changes of hippocampal dysfunction. Abnormal changes in hippocampus are helpful to provide new insights into neuropathological changes in pain-related dysfunction of CTN, which may be helpful for clinical selection of surgical intervention time and provide new ideas and methods for comprehensive treatment of CTN-related complications.

In the future, our research should focus more on the hippocampus subregion, and make a more detailed division of the hippocampus. In addition, the potential dynamic nature of hippocampus structural changes in chronic pain also deserves our attention, and the longitudinal study of hippocampus changes before and after the CTN surgery is also worthy of attention.

The article "Altered Structural and Functional Abnormalities of Hippocampus in Classical Trigeminal Neuralgia: A Combination of DTI and fMRI Study" was published in 2022. Journal: J Healthc Eng.

## Figures and Tables

**Figure 1:** Fractional anisotropy (FA) and apparent diffusion coefficient (ADC) values in the right hippocampus of one patient.

**Figure 2:** ReHo difference between CTN group and HC; correlations between ReHo values and the MOCA score of CTN patients. R: right; L: left.

**Table 1:** Demographic data.

	Age	Side (L/R)	Duration	Carbamazepine dose (g)	VAS score	MOCA score	CDR score
CTN (*n* = 27)	57.6 ± 7.5	14/13	4.95 ± 3.10	1000 ± 800	5.23 ± 2.41	22.26 ± 2.47	0.76 ± 0.25
HC (*n* = 27)	58.1 ± 5.6	—	—	—	0	28.16 ± 1.35	0.18 ± 0.05
*P*	0.81	—	—	—	0.000	0.031	0.000

CTN, classical trigeminal neuralgia; HC, healthy controls; MOCA (Montreal cognitive assessment), VAS (visual analogue scale), CDR (clinical dementia rating).

**Table 2:** The comparison of ADC, FA, and ReHo values in CTN patients and HC.

	CTN patients	Healthy controls	*t*	*P*
ReHo	1.143 ± 0.27	0.976 ± 0.08	2.986 (peak)	0.006
ADC (×10^−3^ mm^2^/s)	0.835 ± 0.09	0.822 ± 0.08	0.640	0.525
FA	0.528 ± 0.06	0.500 ± 0.01	2.387	0.021

**Table 3:** Correlations between ReHo, ADC, FA values and the MOCA, VAS, and CDR scores in CTN patients.

	MOCA	VAS	CDR
	Pearson's correlation (Significance two-tailed)	Pearson's correlation (Significance two-tailed)	Pearson's correlation (Significance two-tailed)
ReHo	0.835(0.000)	0.232(0.195)	0.105 (0.559)
ADC	0.144 (0.423)	0.136 (0.450)	−0.017 (0.927)
FA	0.345 (0.049)	−0.269 (0.130)	−0.019 (0.918)

**Table 4:** Correlations between ReHo values and ADCand FA values of CTN patients.

	Pearson's correlation	Significance (two-tailed)
ReHo and ADC	0.125	0.646
ReHo and FA	0.316	0.234

## Data Availability

The original research data used to support the findings of this study are available from the corresponding author upon request.
